The article "Approaching treatment for immunological rejection of living-donor liver transplantation in rats" was retracted in 2022. Reasons: duplicated images; unreliable data.

# Approaching treatment for immunological rejection of living-donor liver transplantation in rats

**DOI:** 10.1186/s12876-019-1130-x

**Published:** 2020-01-13

**Authors:** Yanhu Feng, Zhijian Han, Zedong Feng, Bofang Wang, Huijuan Cheng, Luxi Yang, Yangbing Li, Baohong Gu, Xuemei Li, Yahao Li, Yumin Li, Chen Wang, Hao Chen

**Affiliations:** 1 Department of Gastroenterology, Lanzhou University Second Hospital, Lanzhou, 730030 China; 2 Key Laboratory of the Digestive System Tumors of Gansu Province, Lanzhou University Second Hospital, Lanzhou, 730030 China; 3 Medical School of Lanzhou University, Lanzhou, 730030 China; 4 Department of Tumor Surgery, Lanzhou University Second Hospital, Lanzhou, 730030 China; 5 Department of General Surgery, Lanzhou University Second Hospital, Lanzhou, 730030 China

**Keywords:** Living donor liver transplantation, Small-for-size syndrome, Tacrolimus, Immunotherapy

## Abstract

**Background:**

The anti-immunological rejection therapy for small-for-size syndrome (SFSS) after live donor liver transplantation (LDLT) play a central role in keeping graft survival. The hepatocyte number and grafts function has undergone real-time changes with the proliferation and apoptosis of the grafts after reperfusion. Lacking an accurate and effective treatment regiments or indicators to guide the use of immunosuppressive drugs in SFS liver transplantation has made immunotherapy after SFS liver transplantation an urgent problem to be solved. Herein, we established small-for-size (SFS) and normal size liver transplantation model in rats to explore the effective indicators in guiding immunotherapy, to find an effective way for overcoming SFSS.

**Methods:**

Lewis rats (donors) and BN rats (recipients) were used to mimic allograft liver transplantation and treated with tacrolimus. Local graft immune response was analyzed through haematoxylin and eosin and immunohistochemistry. Flow cytometry was used to assess the overall immune status of recipient. The pharmacokinetics mechanism of immunosuppressive drugs was explored through detecting CYP3A2 expression at mRNA level and protein levels.

**Results:**

The results showed the local immune reaction of SFS grafts and systemic immune responses of recipient were significantly increased compared with those in normal size grafts and their recipient at four days after liver transplantation. Regression equation was used to regulate the tacrolimus dose which not only controlled tacrolimus serum concentration effectively but alleviated liver damage and improved survival rate.

**Conclusions:**

This study showed that AST level and tacrolimus serum concentrations are effective indicators in guiding immunotherapy. Regression equation (T_D_ = − 0.494T_C_-0.0035AST + 260.487) based on AST and tacrolimus serum concentration can be used as a reference for adjustment of immunotherapy after SFS liver transplantation, which is applicable in clinical practice.

## Background

Living donor liver transplantation (LDLT) has been used as a novel surgical technique for patients with end-stage liver disease since the first successful report in 1990 [1]. Split liver transplantation, LDLT and donation after circulatory death enlarged the organ pool for liver transplantation effectively [2]. These techniques are becoming the options used in therapy from infants to adults to address the shortage of donor organs [3–6]. However, small liver volume is unable to meet the adequate metabolic, synthetic and stably hemodynamic demands of the recipients. The postoperative allograft dysfunction, liver failure and potential severe morbidity or death have been termed as small-for-size syndrome (SFSS) [7]. Studies have shown that recipients also produce stronger immune rejection in the case of small-for-size (SFS) grafts when compared with normal volume liver grafts [8]. Recipients usually require an intensive immunosuppressive regimen, such as tacrolimus, to counter the enhanced rejection. However, severe organ damage and increased side effects (nephrotoxicity, hypertension and neurotoxicity) appeared in a dose-dependent manner [9]. What are the potential mechanisms for the change of tacrolimus metabolic dynamics in SFS liver transplantation? There is no effective and reliable treatment modality for immune rejection after SFS transplantation so far [10]. Graft volume and recipient standard liver volume ratio (GV/SLV) can be used as selection criteria but it only reflects the amount of residual liver cells and it is not representative of the liver function. So GV/SLV has to be assessed together with other factors, such as donor age, severity of the portal hypertension and the Model for End-Stage Liver Disease score of the recipient [11, 12]. Theoretically, the cell number and grafts function has undergone real-time changes with the proliferation and apoptosis of the grafts after reperfusion. Lacking an accurate and effective treatment regiments or indicators to guide the use of immunosuppressive drugs in SFS liver transplantation has made immunotherapy after SFS liver transplantation an urgent problem to be solved. We herein demonstrated the immune rejection change of SFS allograft in rats and explored the drug metabolic characteristic of tacrolimus in vivo in order to develop reliable guidance for immune rejection treatment after SFS transplantation.

## Methods

### Animals and ethics

The protocol of animal experiments was approved by the animal management committee of Lanzhou University Second Hospital and performed strictly according to the guideline on animal experimentation. Adult male Lewis rats and Brown Norway (BN) rats were purchased from Vital River, Beijing with weight 250-260 g and feeding in the standard SPF environment. Lewis rats were used as donors and BN rats as recipients. This method was also used in previous studies to establish allograft immunological rejection in rat liver transplantation model [13].

### Study design

The rat orthotopic liver transplantation model was established based on Kamada’s technique [14]. The Man K technique was implemented for hepatolobectomy to obtain small volume of liver graft in rats [15]. The middle lobe of the donor rat was left untouched, while the other lobe underwent ligation and resection to prepare for transplantation. In the control group, the normal whole liver was used as donor, and the weight of the liver in SFS group was about 40% of the recipient liver (range from 35 to 42%). After abdominal aortic catheterization, the liver is slowly perfused with 8 ml of Ringer’s balanced solution. The portal vein is then transected and the liver taken out. The isolated graft is put in a container filled with ice-cold saline for further preparation. The prosthetic casing is then sheathed outside the portal vein and the infra hepatic vena cava. Portal vein and the infra hepatic vena cava are everted and fixed on the casing. All of the steps were under the good control, no complication was found. Finally, the small size or whole size orthotopic graft is transplanted into the recipient rat. After completion of the surgical procedure, recipient animals were recovered according to an intensive post-operative protocol. The warm ischemia time was 4 ± 1.6 min, the cold ischemia time was 31 ± 2.7 min.

Animals were divided into seven groups: (1) group of whole liver isograft (WI): BN rats as donors and recipients, *n* = 7; (2) group of small-for-size isograft (SI): BN rats as donors and recipients, *n* = 7; (3) group of whole liver allograft (WA): Lewis rats as donors and BN rats as recipients, n = 7; (4) group of small-for-size allograft (SA): Lewis rats as donors and BN rats as recipients, n = 7; (5) group of whole allograft tacrolimus treatment (WAT): Lewis rats as donors and BN rats as recipients, n = 7 (TAC99–25, Tecoland, USA, 1 mg/Kg, intramuscular injection); (6) group of small-for-size allograft tacrolimus treatment (SAT): Lewis rats as donors and BN rats as recipients, n = 7; (7) group of SFS allograft tacrolimus altered treatment (SATa): Lewis rats as donors and BN rats as recipients, n = 7, (TAC99–25, Tecoland, USA. Dosages were adjusted according to the tacrolimus concentration and AST level and given as an intramuscular injection).

The survival of recipient rats was not recorded until death from rejection. In order to obtain the solid and liquid samples, additional three recipient rats of each group were “sacrifice” after reperfusion at different time point. The rats were euthanized by IP injection of Euthanyl Forte (dosage:100 mg/kg, Virbac AH Inc., TX, USA).

Blood samples were taken before the “sacrifice” of the rats and the samples were sent to detect liver function. After the “sacrifice” of the rats, samples were collected including liver, kidney, lung, heart, and stomach. The specimens were also collected if the animal died. The death of the recipient was confirmed by histopathology.

### Tissue processing for haematoxylin and eosin (HE) stain

All liver specimens were fixed by immersion for at least one day in 10% buffered formaldehyde phosphate. The tissues were subsequently dehydrated and embedded in paraffin wax to cut sections and performed HE staining as routine procedure.

### Immunohistochemistry (IHC)

Immunohistochemical staining was performed using a HRP/DAB Detection IHC kit (Abcam, Cambridge, MA, USA) and counterstained with haematoxylin. The primary antibody was αβTCR (1:200 mouse monopoly antibody, Santa Cruz Biotechnology Inc., American) and PCNA (1:250 mouse monopoly antibody, Santa Cruz Biotechnology Inc., America). The results were analyzed by liver cell counting (100 cells per fields for 10 fields were counted for each section, namely about 1000 hepatocytes were counted) and calculating the percentage of αβTCR and PCNA positive cells.

### TUNEL (terminal Deoxynucleotidyl Transferase mediated Nick-end labeling)

Nucleus was counterstained with haematoxylin, mounted with neutral gum and viewed under the microscope. Images shown are representative of at least three independent experiments which gave similar results. The results were analyzed by liver cell counting as PCNA staining.

### Liver function test

The specimens were sent to the second Affiliated Hospital of Lanzhou University where liver function was detected through an automatic biochemical analyzer.

### Western blot

Western blot was performed with general procedure and Gelworks 1D software (UVP, Inc.) was used to analyze the protein expression intensity and calculate the proportion of CYP3A2 protein intensity with β-actin protein intensity in the same samples (CYP3A2abtibody 1:1000 Abcam, catalog number ab195627; β-actin 1:2500, ProteinTech, catalog number 60008–1-Ig). The result was recorded as mean ± SD.

### Statistical analysis

All data are presented as means±SD. Statistical analysis was performed by the t test and Kruskal-Wallis test using SPSS19.0 software. Survival rates were assessed by the Kaplan-Meier method. The log-rank test was used to compare significance. Chi-square test analyzed the positive expression ratio of αβTCR positive staining cells. The CD4 + CD25+ positive cells percentage, liver function, serum blood indexes, IL-17 and CYP3A2 expression levels and tacrolimus serum concentration were analyzed by Student’s t-test or Kruskal–Wallis test. Manmy-whity test and logistical regression analysis were used for correlation analysis. *P* < 0.05 was considered statistically significant.

## Results

### Survival analysis

All recipients of SFS allograft group, the group without immune rejection therapy, died within nine days. Their average survival time was 6.29 days which was lower than the WA group which survived an average of 8.29 days (*P* = 0.027). The use of Tacrolimus significantly prolonged the survival time of the WAT and the SAT groups whose survival time were 57.43 days and 28.00 days respectively, significantly higher than the untreated group (*p* < 0.01). The survival time of the SAT group was lower than the WAT group although they received the same tacrolimus treatment (*p* = 0.047). Compared with the SAT group, the mean survival time for the SATa group was significantly prolonged by adjusting the amount of tacrolimus under the guidance of a regression equation based on tacrolimus blood concentration and AST serum values (39.71 ± 28.99, *p* = 0.331). The 28 days cumulative survival rate of WAT group was 85.7% which was significantly higher than the SAT group of 28.6% (*P* = 0.019, log-rank test). The SATa group’s cumulative survival rate was 51.7% which also higher than the SAT group. But there was no statistical difference (*P* = 0.266, log-rank test) (Fig. 1 and Table 1).

**Fig. 1:** Survival analysis. Tacrolimus remarkably prolonged both WAT and SAT group survivals (*p* < 0.01, compared with WA and SA), but there was still significant difference between WAT and SAT *p* = 0.047). Compared to the SAT group, mean survival time was much longer than that in SATa group (*p* = 0.331). 28-day cumulative survival rates (85.7%) of WAT group were higher than SAT group (28.6%) (*P* = 0.019, log-rank test). The survival rate (51.7%) of SATa is higher than SAT group (*P* = 0.266, log-rank test). whole size allografrs (WA), small-for-size allograft (SA), whole size allografrs+Tac (WAT), small-for-size allograft+Tac (SAT), small-for-size allograft+Tac altered dose (SATa)

**Table 1:** Survival time after liver transplantation

Group	Number	Survival days	Mean + SD
WA	7	7, 7, 8, 8, 8, 9,11	8.29 ± 1.38
SA	7	4, 5, 6, 6, 7, 7, 9	6.29 ± 1.54
WAT	7	25, 30, 45, 60, 63, 89, > 90^*^	57.43 ± 24.97
SAT	7	5, 9, 12, 15, 20, 45, > 90	28.00 ± 29.12
SATa	7	8, 12, 23, 29, 51, 65, > 90	39.71 ± 28.99

^*^>90 was taken as 90 on statistic analysis

### Histological features in liver graft, lungs and kidneys

The whole size liver isograft was normal at four days after reperfusion. The SFS isograft showed morphological changes with moderate red blood cells accumulation in sinus cavity. Large amounts of cell infiltration and some liver structures destruction was present in both whole size and SFS allograft rats. Acute rejection was found in SFS allograft rats including portal area inflammatory cell infiltration, hepatic sinusoidal endothelial cells inflammatory changes, bile duct necrosis and hepatic sinusoid cells infiltration (Fig. 2). The pathological damage to lungs and kidneys was more obvious in the SAT group four days after surgery including pulmonary interstitial edema, lymphocyte infiltration, erythrocyte exudation, alveolar wall thickening, progressive glomerular swelling and diffuse nephrolithia ball-like bleeding. All of the above-mentioned organ pathological lesions were significantly reduced or did not occur in the SATa Group (Fig. 2).

**Fig. 2:** Histology of liver grafts and other organs at four days after transplantation. HE staining magnification × 120, whole size allografrs+Tac (WAT), small-for-size allograft+Tac (SAT), small-for-size allograft+Tac altered dose (SATa). Whole size isograft (WI), small-for-size isograft (SI), whole size allograft (WA), small-for-size allograft (SA)

### Infiltrating lymphocytes phenotypic of liver graft and detection of hepatocyte proliferation and apoptosis

Immunohistochemical analysis showed that the αβTCR positive lymphocytes in allografts were significantly higher than that of the isografts at four days after transplantation. Similarly, the αβTCR positive expression cell number in SFS allografts was significantly higher than that in whole size allografts (*p* < 0.05, Fig. 3).

**Fig. 3:** αβTCR staining and proliferation and apoptosis detection. αβTCR were the main population of infiltrating cells in SFS allografts at four days after operation. The ratio of αβTCR cells was higher in SFS allograft than in whole size allograft. SAT and SATa groups showed increased hepatocyte proliferation and apoptosis compared with WAT group 4 days after operation, which characterized by higher PCNA expression and more positive cell by TUNEL (*P* < 0.01). Immunohistochemical staining magnification × 120, whole size allografrs+Tac (WAT), small-for-size allograft+Tac (SAT), small-for-size allograft+Tac altered dose (SATa). Whole size isograft (WI), small-for-size isograft (SI), whole size allograft (WA), small-for-size allograft (SA)

Compared with the WAT group, the proportions of PCNA positive expression and TUNEL positive staining were significantly increased in the SAT and the SATa group (*P* < 0.01). The hepatocytes proliferation was significantly increased in the SATa group compared with the SAT group (p < 0.05). On the contrary, the number of apoptotic cells was significantly decreased (*p* < 0.05) (Fig. 3).

### Phenotypic analysis of peripheral blood lymphocytes in recipients

Flow cytometry showed that CD4 + CD25+ lymphocytes were significantly less in peripheral blood of allografts than isografts four days after transplantation. Similarly, the positive expression rates of CD4 + CD25+ lymphocytes in SFS allografts was significantly lower than those in whole size allografts (*p* < 0.01, Fig. 4).

**Fig. 4:** CD4^+^CD25^+^ number and hepatocyte proliferation and apoptosis in SFS allograft were changed four days after operation. Flow cytometry analysis of phenotypic peripheral lymphocytes showed a dramatic decrease in CD4 + CD25+ cells in allograft recipient compared with that in isograft recipient(*P* < 0.05). The decrease was greater in the SFS allograft recipient than in the whole size allograft recipient (*p* < 0.01)

### Expression of cytokine IL-17 and CYP3A2

IL-17 was hardly expressed in isografts four days after the operation. The expression of IL-17 was increased by three times in whole size allografts and five times in SFS allografts in comparison with the corresponding isografts (P < 0.01). Its expression in SFS allograft was also significantly higher than that in whole size allografts (*P* < 0.05, Fig. 5).

**Fig. 5:** Expression of IL-17 and CYP3A2. **a** Increased IL-17 expression was observed in SFS allograft four days after operation. **a**) IL-17 expression was significantly enhanced in allograft, three folds in WA group and five folds in SA group compare to the WI and SI group (p < 0.01). **b**, **c**) Expression of CYP3A2 was significantly decreased in small-for-size live transplantation at postoperative early period. CYP3A2 expression level was on a apparent decline of about 60% at 12 h, 50% at 24 h, 30% at 48 h (*p* < 0.05) after transplantation in SA group compare to WA group. However, CYP3A2 expression level was gradually recovered by 96 h. Whole size isograft (WI), small-for-size isograft (SI), whole size allograft (WA), small-for-size allograft (SA)

The expression of CYP3A2 decreased significantly in the early postoperative period for SFS liver grafts. Compared with the normal size whole liver transplantation group, the expression of CYP3A2 in SFS grafts decreased by about 60% at 12 h, 50% for 24 h and 30% for 48 h after transplantation. However, the expression of CYP3A2 gradually recovered at 96 h after transplantation (Fig. 5).

### Tacrolimus blood concentration analysis

The blood concentration of tacrolimus was significantly higher in the SFS transplantation with tacrolimus routine treatment group than the whole size transplantation group at different time points (*p* < 0.05). The peak concentration of tacrolimus in the SFS group was more than two times higher than the whole size transplantation group. However, the tacrolimus blood concentration was relatively stable in SFS group after adjusting the dosage of tacrolimus under the guidance of the regression equation based on tacrolimus blood concentration and AST level. Moreover, the serum concentration of tacrolimus was significantly lower in the SFS group using altered dose on the basis of Tc and AST (SATa) than that of the unadjusted SFS group (SAT) (*P* < 0.05, Fig. 6).

**Fig. 6:** Increased Tac blood concentration in SAT group and recovered Tac blood concentration in SATa (*n* = 3 each group). Compared with WAT group, Tac blood concentration was increased in SAT group after operation (p < 0.05). However, Tac blood concentration kept stable in SATa group after operation and Tac level was significantly lower in SATa group than SAT group at 24, 48, and 72 hs after operation (P < 0.05). AST and bilirubin concentration increased dramatically in SAT and SATa group after operation (n = 3 each group). Compared with WAT group, AST concentration in SAT and SATa group increased dramatically during 48hs after operation (p < 0.01). AST concentration was lower in SATa group than WAT group although there was no significant difference between WAT and WATa groups. Whole size allografrs+Tac (WAT), small-for-size allograft+Tac(SAT), small-for-size allograft+Tac altered dose (SATa)

### Liver function analysis

Compared with the WAT group, AST concentration were significantly higher in SAT group and SATa group 48 h after operation (*p* < 0.01). The AST concentration of the SATa group was lower than the SAT group although there was no significant difference statistically between SAT group and SATa group. The trend of total bilirubin was similar to AST (Fig. 6).

### Correlation analysis

The changes in serum concentration of tacrolimus and the corresponding values of RCA (ratio of CYP3A4 to actin), RPA (ratio of proliferation to apoptosis) and AST are listed in Table 2. Correlation analysis showed a significant correlation between RCA, RPA, and AST (RCA and RPA R = 0.976 *P* = 0.001; RPA and AST R = − 0.962 P = 0.001; RCA and AST R = -0.906 *P* = 0.005). The serum concentration of tacrolimus decreased with the decrease of AST (R = 0.758 *P* = 0.046). The Logistical regression equation was TD = − 0.494TC-0.0035AST + 260.487 (Fig. 7).

**Table 2:** Changes in tacrolimus blood concentration (Tc) and RCA, RPA, AST after liver transplantation

	0.5d	1d	2d	3 d	4d	5d	6d
RCA	0.269 ± 0.030	0.310 ± 0.021	0.452 ± 0.015	0.590 ± 0.041	0.621 ± 0.053	0.756 ± 0.049	0.789 ± 0.056
RPA	0.76 ± 0.089	0.88 ± 0.098	1.39 ± 0.01	4.8 ± 0.14^*^	5.2 ± 0.25	6.5 ± 0.36	6.9 ± 0.49
AST	895.1 ± 168.8	1186.6 ± 378.2	1120.5 ± 298.5	599.1 ± 277.7^*^	419.9 ± 201.2	227.6 ± 140.9	189.1 ± 110.3
T _C/D_	10.03 ± 1.15	11.46 ± 1.59	13.58 ± 2.01	12.21 ± 2.68	10.89 ± 2.35	8.01 ± 1.98	6.16 ± 1.24

^*^P < 0.01 versus 2 days, RCA (Ratio of CYP3A4 to actin), RPA(Ratio of proliferation to apoptosis), AST(asparatate aminotransferase), T_C/D_ (tacrolimus blood concentration/dose ratio)

**Fig. 7:** Correlation analysis. A significant correlation was found between RCA, RPA and AST (RCA and RPA R = 0.976 *P* = 0.001; RPA and AST R = − 0.962 P = 0.001; RCA and AST R = -0.906 *P* = 0.005). The tacrolimus blood concentration was decreased as AST (R = 0.758 *P* = 0.046). Logistical regression analysis shows regression equation: T_C_ = 0.005AST + 7.223, T_D_ = − 0.007AST + 257.757, T_D_ = − 0.988TC + 263.219; T_D_ = − 0.494T_C_-0.0035AST + 260.487. RPA (Ratio of proliferation to apoptosis), AST (asparatate aminotransferase), Tc (tacrolimus concentration), T_D_ (tacrolimus dose)

## Discussion

SFS liver transplantation as an effective means of expanding the donor liver has been recognized worldwide. Although the successful implementation of surgical techniques has resulted in a significant reduction in the mortality rate of patients waiting for liver transplantations, the surgery itself inevitably leads to new compelling problems related to the difficulty in immunotherapy after SFS liver transplantation.

Although the optimal size of grafts for SFS liver transplantation remains the focus of controversy, it is generally assumed that the graft-to-recipient weight ratio should exceed 0.8% and GV/SLV should exceed 35–40%. According to the Fan [16] and Kawasaki [17] proposed guidelines, the volume fraction of small grafts was chosen 40% (35–42%) in our study. In order to explore whether recipients drive different degrees of rejection as the graft volume changes, animal models of the whole liver volume and SFS allograft and isograft were established and the rejection between them were compared. The results showed that acute rejection was more pronounced in SFS grafts (Fig. 2). A large number of inflammatory cells infiltrated into hepatic sinus and around the portal area. These infiltrating inflammatory cells were dominated by αβTCR positive phenotypes, which indicated that the infiltrating cells were mature lymphocytes. αβTCR plays an important role in antigen presentation. Expression of αβTCR on lymphocytes contributes to the enhancement of immune responses (Fig. 3). In addition to the enhanced local immune response, the systemic immune response was also significantly strengthened in SFS transplant recipients, and the number of CD4 + CD25 + T lymphocytes in peripheral blood was decreased significantly (Fig. 4) while the expression level of IL-17 increased significantly (Fig. 5).

CD4 + CD25 + T cells can inhibit the activation, proliferation and function of T lymphocytes [18]. CD4 + CD25+ T cells also inhibited allograft T lymphocyte responses. For example, it suppresses allograft rejection of the skin and solid organs [19–21]. Studies have shown that CD4 + CD25+ T cells play a key role in immune tolerance models [22, 23]. Recent studies found IL-17 levels were increased in acute rejection of animal models or patients after early transplantation of the kidneys, lungs and heart [24–26]. In our study, the elevated expression of IL-17 was observed in an acute rejection model of SFS liver transplantation in rats. The above evidence suggests that the recipient has enhanced immune rejection of SFS allografts. This is consistent with the Takashi Omura study [27].

Tacrolimus is metabolized predominantly in the liver as most of the immunosuppressive drugs. However, the number of hepatocytes reduced due to the SFS surgery and liver function was impaired after ischemia-reperfusion, therefore, the metabolic capacity of hepatocytes was inevitably affected to some extent. As a result, the plasma concentration of tacrolimus was likely to increase in the case of reduced hepatocyte metabolism in SFS liver grafts. To prove the hypothesis, the plasma concentration of tacrolimus was measured at different time points after the whole size and SFS liver transplantation (Fig. 6). High concentrations of tacrolimus not only aggravated liver metabolic burden, but also caused other organs damage as well as unpredictable side effects. In the early stage of transplantation, the concentrations of AST and total bilirubin in the SFS recipients were increased significantly compared with the normal size liver transplant recipients, and the number of apoptotic cells was also increased significantly (Fig. 6). Organs damage would inevitably affect the survival rate of grafts and recipients. Although tacrolimus can significantly prolong the survival in the normal size and SFS recipients compared with the subjects without using tacrolimus (*p* < 0.01), the average survival time of the SFS graft was significantly lower than that of the normal size liver graft (*p* = 0.047).

The mechanism under the change in tacrolimus blood concentration was explored to find an effective way to accurately guide tacrolimus use for SFS graft recipients. Cytochrome P450 3A enzymes play a central role in the metabolism of almost 50% of the currently used drugs including tacrolimus [28]. In particular, Ca-neuromycin inhibitors are mainly metabolized by the CYP3A4 enzyme, which is a metabolic enzyme in the liver. The CYP3A4 enzyme in the human liver is equivalent to the CYP3A2 enzyme in the rat liver [29, 30]. In our previous study, we showed that cytochrome oxidase CYP3A and drug efflux pump P-gp were two major influencing factors in drug metabolism. The polymorphisms of P-gp and CYP3A were found to be closely related to tacrolimus plasma concentrations among different individuals [31]. Our current study found that the expression of CYP3A2 was significantly reduced in the early stages of SFS grafts. The results were similar to those of Powis and his colleagues, who found that the content and activity of CYP3A4 rapidly decreased after partial resection of human liver [32]. However, molecular mechanism how the graft volume change affecting the CYP3A2 will be further elucidated in subsequent studies. We have already discovered that nitric oxide signaling pathways potentially play an important role in this mechanism.

The ratio of hepatocyte proliferation and apoptosis (RPA) significantly increased when the CYP3A2 level gradually recovered 72 h after transplantation (*p* < 0.01). Correlation analysis was performed in order to find the relationship between CYP3A2, RPA and AST. RPA represents the SFS liver graft regeneration capacity, which increases with hepatocytes proliferation and decrease of apoptosis. After SFS liver transplantation, surviving small-volume grafts tend to proliferate to the original liver volume. Drug metabolism capacity was also enhanced as hepatocytes number increased and the liver function was restored. As shown in this study, CYP3A2 increased as RPA increases. AST decreased with the recovery of liver function which was consistent with the results. RPA was negatively correlated with AST.

Many attempts have been made to find a method for the treatment of immune rejection after SFS liver transplantation. Kishino and his colleagues showed that the CYP3A4 difference between individuals was caused by graft volume and recipient liver standard volume ratio and the recipient age [33]. In addition, Fukatsu et al. reported that there was a significant correlation between the weight of the graft and the clearance of tacrolimus in patients receiving liver transplantation [34]. Sugawara’s study indicated that there was a correlation between the optimal dose of tacrolimus and GV/SLV. The dose of tacrolimus early after SFS liver transplantation could be estimated by using the equation established by the GV/SLV [35].

## Conclusions

In summary, a regression equation was established based on logistic regression analysis of tacrolimus plasma concentration and AST (T_D_=− 0.494T_C_-0.0035AST+260.487). The dose of tacrolimus was adjusted based on this equation in the early postoperative period in rats. More importantly, blood specimens are easier to obtain. Therefore, it is an effective and feasible method to adjust the dose of tacrolimus after SFS liver transplantation using our established regression equation. There are also shortcomings in this experiment. Although the tacrolimus is the main drug to anti-rejection in clinical practice, other drugs need to be tested in the future. Clinical trials are needed to further evaluate the value of this study in immunotherapy for SFS liver transplantation. CYP2C, which has a role closer to human CYP3A enzymes did not be measure, will be tested in ongoing study.

## Abbreviations

AST: Aspartate aminotransferase
BN rats: Brown Norway rats
CYP3A2: Cytochrome P450 3A2
GV/SLV: Graft volume and recipient standard liver volume ratio
IHC: Immunohistochemistry
LDLT: Live donor liver transplantation
PCNA: Proliferating cell nuclear antigen
RCA: Ratio of CYP3A4 to actin
RPA: Ratio of proliferation to apoptosis
SFS: Small-for-size
SFSS: Small-for-size syndrome
TUNEL: Terminal deoxynucleotidyl transferase dUTP nick end labeling
